# Fasting Whole Blood Fatty Acid Profile and Risk of Type 2 Diabetes in Adults: A Nested Case Control Study

**DOI:** 10.1371/journal.pone.0097001

**Published:** 2014-05-09

**Authors:** Amani Alhazmi, Elizabeth Stojanovski, Manohar L. Garg, Mark McEvoy

**Affiliations:** 1 Nutrition and Dietetics, School of Health Sciences, Faculty of Health and Medicine, University of Newcastle, NSW, Australia; 2 Ministry of Higher Education, Riyadh, Saudi Arabia; 3 School of Mathematical and Physical Sciences, Faculty of Science and Information Technology, University of Newcastle, NSW, Australia; 4 School of Biomedical Sciences & Pharmacy, Faculty of Health and Medicine, University of Newcastle, NSW, Australia; 5 Centre for Clinical Epidemiology & Biostatistics, Faculty of Health and Medicine, University of Newcastle, NSW, Australia; Oklahoma State University, United States of America

## Abstract

**Objective:**

to determine the association of fasting whole blood fatty acid concentrations with incidence of type 2 diabetes in adults.

**Methods:**

A nested case-control study of 187 subjects from a cohort of men and women aged 55–85 years from the Hunter Region, New South Wales, Australia. Fasting whole blood fatty acids were measured using gas chromatography and incidence of type 2 diabetes was ascertained by self-reported questionnaire at the study follow-up.

**Results:**

After adjustment for potential confounding variables, positive associations with type 2 diabetes were seen for dihomo-gamma-linolenic acid (DGLA) (OR = 1.04, 95% CI:1.01–1.07, *P* = 0.01); arachidonic acid (ARA) (OR = 1.01, 95% CI:1.00–1.01, *P* = 0.002); alpha-linolenic acid (ALA) (OR = 1.10, 95% CI: 1.03–1.18, *P* = 0.01); eicosapentaenoic acid (EPA) (OR = 1.05, 95% CI:1.02–1.08, *P* = 0.001); and docosahexaenoic acid (DHA) (OR = 1.03, 95% CI:1.02–1.05, *P*<0.0001). Lignoceric acid is significantly associated with lower type 2 diabetes risk (OR = 0.95, 95% CI: 0.92–0.99, *P* = 0.01).

**Conclusion:**

These data suggest that higher fasting whole blood concentrations of omega-6 polyunsaturated fatty acids (n-6PUFA) (ARA and DGLA) as well as omega-3 polyunsaturated fatty acid (n-3PUFA) (ALA, EPA, and DHA) are associated with an increased risk of diabetes, whereas increased fasting whole blood concentrations of lignoceric acid is inversely associated with diabetes risk.

## Introduction

Diabetes, mostly in the form of type 2, has become both an economic and health problem globally [1]. The prevalence of diabetes among the adult population worldwide is 285 million, and is expected to increase to 439 million by 2030 [2]. Since type 2 diabetes is associated with significant comorbidity and increased mortality, strategies to prevent the development of type 2 diabetes is the ideal approach to reduce the burden of this disease. Environmental and lifestyle factors such as diet are well established modifiable contributors to the development of type 2 diabetes. Results from recent epidemiological studies suggest that dietary fatty acid intake may be among the most critical dietary factors that influence the development of type 2 diabetes [3], [4], [5], [6].

Despite the tremendous interest in elucidating the relationship between dietary fat and type 2 diabetes, the evidence remains limited by the inaccuracy of fatty acid assessment methods. Most existing studies have relied on dietary questionnaires to estimate fatty acid consumption [7], [8], [9], [10], which may be prone to a measurement error of habitual fat intake. The use of quantitative measurements of individual fatty acids in blood is particularly desirable because it provides an objective measure of exposure that may represent an unbiased estimate of fatty acid reserves. A few epidemiological studies have measured fatty acids in plasma or serum and examined these concentrations in relation to the development of type 2 diabetes [3], [11], [12], [13], [14]. Plasma and serum however, reflect fatty acid composition of dietary fat consumed in the previous 24 hours [15] but are not reliable indicators of long–term status or the usual intakes. A previous study showed that fasting whole blood is a suitable biomarker of fatty acid intake [15]. However, studies reporting its association with type 2 diabetes incidences are lacking. Given the inconsistencies of the evidence examining the association of fatty acid intake with incident type 2 diabetes and the inaccuracy of the methods used to measure fatty acid status, the aim of this study was to use a nested case-control design to determine the association of fasting whole blood fatty acid concentrations with incidence of type 2 diabetes in adults.

## Materials and Methods

### Study population

Participants for the current investigation were derived from the Hunter Community Study (HCS), which is a population-based cohort study of men and women aged 55–85 years living in the Hunter Region, NSW. Detailed descriptions of sampling, recruitment, and methods employed by these studies can be obtained from its baseline descriptive paper [16]. Briefly, the HCS was designed to assess a range of bio-psychosocial aspects of ageing. Participants were randomly selected from the NSW State Electoral Roll and contacted between mid-December 2004 and June 2005. A recruitment strategy was used whereby two letters of introduction were posted to the selected persons, with a follow-up phone call. If contact was not established after five attempts, the individual was classified as a non-responder. Those who could not speak English were deemed ineligible. Once written informed consent to participate was obtained, eligible individuals were asked to provide a blood sample, complete a series of self-report postal questionnaires, and receive a clinical assessment. Consent to link data from Medicare Australia (Medicare and Pharmaceutical Benefit Scheme) with local health databases was also obtained.

Follow-up of the cohort occurred in 2011; 3318 participants were sent a follow-up postal questionnaire that asked about health outcomes and lifestyle factors. By follow-up, the study team was notified of 132 deaths (4%), 169 people actively withdrew (5%) and 767 (23%) were lost to follow-up with unknown reasons, leaving 2250 who completed follow-up questionnaires (response rate = 74%). Those who completed follow-up were significantly younger, more likely to be married and less likely to be widowed, yet had the same gender profile as those who did not complete follow-up. Written informed consent was obtained. The study was approved by the University of Newcastle and Hunter New England Human Research Ethics Committees, NSW, Australia.

### Case and control ascertainment

A self-administered questionnaire was used to ascertain all HCS 5-year incident cases of type 2 diabetes. This questionnaire asked HCS participants if they had ever had a diagnosis of type 2 diabetes and at what age. To ensure that all cases were incident cases of type 2 diabetes any subject with self-reported diagnosis of type 2 diabetes at baseline or fasting serum glucose ≥7.0 mmol/L were excluded from the study. The type 2 diabetes cases for the current investigation were all cases with fasting whole blood available for the determination of fatty acid concentrations (N = 37). Controls were a random sample of the remaining cohort who were not type 2 diabetes cases at follow-up and had a blood sample available (N = 150). The controls sample size was chosen to maximize statistical power (1∶4).

#### Blood collection and fasting whole blood fatty acid measurement

Blood was collected in EDTA tubes and stored at −80°C for fatty acid analysis. There were no previous freeze-thaw cycles. A comprehensive range of fatty acids were analysed by gas chromatography (GC) following methods of Lepage and Roy (1986) [17]. Fatty acid methyl esters (FAME) were separated and quantified using a Hewlett-Packard 6890 and GC equipped with a 30 ml (0.25 mm ID) carbon-silica capillary column coated with 50% cyanoproylphenyl and 50% dimethylpolysiloxane (0.25 µm film thickness), a flame ionisation detector, auto sampler and auto detector. Chemstation version A.04.02 was used for GC analysis and fatty acid methyl esters were identified based on retention time compared to lipid standards and calculated to provide concentration (mg/L).

### Measurement of potentially confounding variables

Age, gender, body mass index (BMI), alcohol intake, smoking, physical activity, supplement use, and dietary intake were considered potentially confounding variables and adjusted for in the analyses by their inclusion in the models as predictors. BMI was calculated as weight (kg) divided by height (m)^2^. Health behaviours including alcohol intake (g/day), smoking status (ever smoke %), and physical activity were consider in the analysis. Step counts were obtained using a Yamax Digiwalker SW-200 pedometer (Yamasa Tokei Keiki Co Ltd, Tokyo, Japan) worn by participants for seven days. The mean daily step count was used as a marker of physical activity. Dietary intake was derived from a single self-administered, previously validated [18], semiquantitative food questionnaire at baseline. Nutrient intakes were determined using a custom-made nutrient analysis programme based on NUTTAB 2006 database [19]. Total intake of energy (kJ), total carbohydrate (g/day), total protein (g/day), fibre (g/day), and supplement use (including fatty acids) (%) were also considered as potential confounding variables.

### Statistical analysis

All analyses were carried out using SAS Version 9.2 (SAS institute, NC, USA). Baseline characteristics of patients were compared between the case and control groups using chi-square tests for categorical variables; and *t*-tests or non-parametric Wilcoxon rank-sum tests for characteristics with highly skewed distributions for numerical variables. For the primary outcome (type 2 diabetes), the odds ratio (OR) and 95% confidence intervals are reported for each group. Three models were created for each fatty acid of interest. Model one was the unadjusted model. Model two adjusted for age in years, and gender. Model three additionally adjusted for physical activity, alcohol intake, smoking status, supplements use, protein, fibre, carbohydrates, and BMI. For the final reported model, independent variables that were not statistically significant were removed using a backward stepwise logistic regression procedure. The associated regression coefficients reflect the relationship between the incidence of diabetes and the corresponding explanatory variables adjusted for total energy intake using the residual method described by Willet and Stampfer [20]. The fit of each multivariable logistic regression model was assessed using Hosmer and Lemeshow's goodness-of-fit test while Akaike's information criterion (AIC) was used to compare models. *T*-tests were performed to assess the association between diabetes status at follow-up and fasting whole blood fatty acids ratios: 18∶1/18∶0, 20∶4n-6/20∶3n-6, 20∶4n-6/18∶2n-6, 22∶6n-3/22∶5n-3, and 22∶6n-3/18∶3n-3. To adjust for the fact that multiple tests were performed, a false discovery rate approach of 0.05 was used [21]. The false discovery rate approach controls the proportion of false positives among the set of tests with statistically significant results.

## Results

Baseline characteristics of the study sample according to type 2 diabetes status are presented in Table 1. Participants in the HCS population who subsequently developed type 2 diabetes had significantly greater BMI and were more likely to be obese at baseline than those who remained diabetes free. Furthermore, participants who developed diabetes had a significantly higher consumption of carbohydrate and protein compared with control subjects.

**Table 1:** Baseline characteristics of the study population (n = 187) from the Hunter community study.

Characteristic	Cases (37)	Control (150)	*P-*value
Age (year)	64.0 (11.0)	65.0 (11.0)	0.20
Gender			
Male (%)	56.76	49.33	0.42
Female (%)	43.24	50.67	
BMI (kg/m2)	30.23 (8.6)	28.15 (5.57)	0.004
Physical activity (Steps-mean)	5548 (3455)	6297.0 (4986)	0.90
Energy (kJ)	8529.050 (4162)	8109 (3285)	0.09
Alcohol intake (g)	0.00 (0.178)	0.00 (0.089)	0.79
Smoking status (%)	34	47	0.18
Using Supplements (%)	25	75	0.07
Carbohydrate (g)	253.65 (125.87)	223.06 (103.09)	0.04
Fibre (g)	32.98 (12.39)	29.58 (12.59)	0.12
Protein (g)	93.80 (42.69)	87.16 (36.17)	0.03
Total fat (g)	67.66 (33.37)	64.68 (30.13)	0.76
Total MUFA (g)	22.68 (9.52)	20.98 (11.15)	0.75
Total PUFA (g)	9.36 (5.47)	9.19 (6.55)	0.72
Total SFA (g)	25.48 (14.96)	24.48 (13.69)	0.86

Values are expressed as median (interquartile range) for continuous variables and percentages for categorical variables.

*P*-values were derived using *t*-tests for continuous variables or the Wilcoxon rank-sum tests for continuous variables displaying significant departures from normality; or the chi-square test for categorical variables.

Abbreviation: BMI, body mass index; MUFA, monounsaturated fatty acid; PUFA, polyunsaturated fatty acid; SFA, saturated fatty acid.

Unadjusted and adjusted logistic regression analyses of fasting whole blood fatty acid concentrations with incidence of type 2 diabetes are reported in Table 2. In the unadjusted logistic regression analyses (Model 1), arachidonic acid (ARA) (C20∶4n-6), dihomo gamma-linolenic (DGLA) (C20∶3n-6), alpha-linolenic acid (ALA) (C18∶3 n-3), eicosapentaenoic acid (EPA) (C20∶5n-3), and docosahexaenoic acid (DHA) (C22∶6n-3) were all statistically significantly associated with type 2 diabetes risk. In the adjusted multivariable logistic regression analyses (Model 3), higher concentration of fasting whole blood DGLA was significantly associated with increased risk type 2 diabetes (OR = 1.04, 95% CI: 1.01–1.07, *P* = 0.01). Increased ARA concentration was also associated with an increased risk of type 2 diabetes (OR = 1.01, 95% CI: 1.00–1.01, *P* = 0.002). Similarly, increased ALA concentration was associated with an increased risk of type 2 diabetes (OR = 1.10, 95% CI: 1.03–1.18, *P* = 0.01). A similar positive association was also observed between EPA and DHA with risk of type 2 diabetes (OR = 1.05, 95% CI: 1.02–1.08, *P* = 001; OR = 1.03, 95% CI: 1.02–1.05, *P*<.0001 respectively). Higher concentration of fasting whole blood lignoceric acid is significantly associated with lower type 2 diabetes risk (OR = 0.95, 95% CI: 0.92–0.99, *P* = 0.01).

**Table 2:** Odds ratios (and 95% CIs) for incident diabetes by fasting whole blood fatty acids, Hunter Community Study.

Fatty acids	Model 1			Model 2			Model 3			AIC; H&L
	OR	95% CI	*P-*value	OR	95% CI	*P-*value	OR	95% CI	*P-*value	
*MUFA*										
OLA (C18∶1n-9)	1.001	1.00–1.003	0.15	1.001	1.00–1.00	0.60	1.00	1.00–1.00	0.13	181;0.30
Palmitoleic acid (16∶1n-7)	1.002	0.99–1.011	0.68	1.00	0.99–1.01	0.48	1.00	0.99–1.01	0.52	171; 0.12
Vaccenic acid (18∶1 n−7)	1.01	0.99–1.03	0.49	1.01	0.99–1.03	0.26	1.01	0.99–1.04	0.19	171; 0.08
Nervonic acid (24∶1n-9)	1.02	0.98–1.04	0.09	1.02	0.99–1.04	0.09	1.02	1.00–1.04	0.12	171; 0.82
*SFA*										
PAM (16∶0)	1.000	0.91–1.00	0.51	1.00	0.99–1.00	0.63	1.00	1.00–1.00	0.34	171; 0.02
STA (18∶0)	1.00	0.91–1.01	0.61	1.00	0.99–1.00	0.73	1.00	1.00–1.00	0.27	171; 0.33
Lignoceric acid (24∶0)	0.96	0.93–0.99	0.008	0.95	0.92–0.98	0.002	0.95	0.92–0.99	0.01	181; 0.87
*n-6 PUFA*										
LNA (18∶2n-6)	1.001	0.99–1.003	0.18	1.00	1.00–1.00	0.11	1.00	1.00–1.01	0.06	171; 0.32
DGLA (20∶3n-6)	1.04	1.01–1.06	0.007	1.04	1.01–1.07	0.004	1.04	1.01–1.07	0.01	181; 0.79
ARA (20∶4n-6)	1.005	1.00–1.01	0.01	1.01	1.00–1.01	0.003	1.01	1.00–1.01	0.002	181; 0.53
*n-3 PUFA*										
ALA (18∶3 n-3)	1.08	1.02–1.14	0.01	1.09	1.02–1.15	0.01	1.10	1.03–1.18	0.01	171; 0.83
EPA (20∶5n-3)	1.03	1.03–1.01	0.02	1.04	1.01–1.07	0.005	1.05	1.02–1.08	0.001	181; 0.37
DHA (22∶6n-3)	1.02	1.01–1.04	<0.001	1.03	1.02–1.04	<.001	1.03	1.02–1.05	<.0001	181; 0.75
DPA (22∶5 n-3)	0.98	0.96–1.01	0.15	0.99	0.97–1.02	0.71	0.99	0.97–1.02	0.58	181; 0.49

Model 1 Unadjusted model.

Model 2 additionally adjusted for age and gender.

Model 3 additionally adjusted for BMI; physical activity; alcohol intake; smoking; supplement use, carbohydrate, fiber, and protein.

Abbreviations: IC, Akaike's information criterion test; ALA, alpha-linolenic acid; ARA, arachidonic acid; DGLA, dihomo-gamma-linolenic acid; DHA, docosahexaenoic acid; DPA, docosapentaenoic acid; EPA, eicosapentaenoic acid; H&L, Hosmer and Lemeshow's goodness-of-fit test; LNA, linoleic acid; MUFA, monounsaturated fatty acids; N-3PUFA, omega-3 polyunsaturated fatty acid; N-6PUFA, omega-6 polyunsaturated fatty acid; OLA, oleic acid; PAM, palmitic acid; STA, stearic acid.

All models fit the data well based on the associated Hosmer and Lemeshow statistics (*P*>0.1). Comparison of each final fatty acid model using the AIC statistic indicates the models with DHA and EPA are the best fitting as they have the smallest AIC (Table 2). Explorative t-tests results showed no significant differences for each of the fasting whole blood fatty acid ratios in cases and controls (Table 3).

**Table 3:** Fatty acid desaturase products in fasting whole blood of type 2 diabetes cases compared with control,Hunter community study^1.^

Desaturase	Fatty acid product/substate	Cases (37)	Control(150)	*P*-value
Δ9	18∶1/18∶0	1.27(0.53)	1.129(0.472)	0.19
Δ5	20∶4n-6/20∶3n-6	5.27 (2.34)	5.11(2.34)	0.32
Δ5, Δ6 (step 1)	20∶4n-6/18∶2n-6	0.44(0.25)	0.41(0.17)	0.30
Δ6	22∶6n-3/22∶5n-3	2.20 (0.99)	1.00 (1.46)	0.75
Δ5, Δ6 (step 1, 2)	22∶6n-3/18∶3n-3	7 (5.93)	6 (6.03)	0.62

1 Data are shown as median (interquartile range).

Abbreviations: 18∶0, Stearic acid; 18∶1, oleic acid; 18∶3n-3, linolenic acid; 20∶3n-6, cis 8,11,14 eicosatrienoic acid; 20∶4n-6, arachidonic acid; 22∶5n-3, cis 7,10,13,16,19 docosapentaenoic acid; 22∶6n-3, cis 4,7,10,13,16,19 docosahexaenoic acid.

## Discussion

This observational population-based nested case-control study examined the association of fasting whole blood fatty acid concentrations with incidence of type 2 diabetes. In unadjusted analyses, increased DGLA, ARA, ALA, EPA, and DHA concentrations were all statistically significantly associated with increased risk of type 2 diabetes. After adjusting for potentially confounding variables, these fatty acids remained statistically significant independent predictors of type 2 diabetes risk. The results also suggested that Lignoceric acid may have a protective function. Direct comparisons between previous studies and the current study are complex due to the use of different biomarkers to determine fatty acid status, using survey and food frequency questionnaire method as opposed to quantitative (e.g. GC used in this study) assessment methods, and population differences in age, sex, lifestyles, and other factors may also affect the associations.

Although the pathogenesis of type 2 diabetes is thought to be related to pro-inflammatory mechanisms [22], DGLA, which is metabolized to the anti-inflammatory eicosanoid, prostaglandin (PG) E_1_, via the cyclooxygenase (COX) pathway [23], was positively associated with type 2 diabetes risk in the current study. However, the DGLA is an extremely uncommon fatty acid and found only in trace amounts in animal products; hence although there is a statistically significant difference between type 2 diabetes cases and controls the small increase in DGLA observed in type 2 diabetes cases in this study may not be clinically relevant.

Evidence is underrepresented regarding the associations between n-6 PUFA, in particular, ARA and type 2 diabetes risk. ARA is known to be metabolized by COX enzymes to produce 2-series prostaglandins, leukotriene, and other bioactive products [24], [25]. These eicosanoids along with elevated levels of pro-inflammatory cytokines, are implicated in the pathogenesis of diabetes mellitus [26]. In contrast with the current finding, the Melbourne Collaborative Cohort Study which included adults aged 36–72 year, reported that plasma ARA were not associated with type 2 diabetes risk [13].

Positive association between the fasting whole blood ALA and type 2 diabetes risk is in agreement with the Melbourne Collaborative Cohort Study, which showed a positive association between plasma phospholipid ALA and type 2 diabetes risk before controlling for BMI [13]. These data also confirm our recent observation that dietary ALA is associated with a higher risk of type 2 diabetes in mid-age Australian women [27]. Another study, however, showed that a higher concentration of plasma ALA is associated with a lower risk of type 2 diabetes in men and women [3]. Compared with fasting whole blood, the use of plasma/serum fatty acids as a biomarker of long-term fatty acid intake has met criticism [28], [29], [30]. Given that type 2 diabetes often develops slowly, over a period of years it is important to consider biomarkers of long-term dietary fatty acid intake. Plasma fatty acid concentrations change rapidly during the day depending on metabolic status and recent dietary intake and are therefore not reliable indictors of long-term fatty acid intake compared with fasting whole blood fatty acid measurements. Epidemiological studies assessing associations between EPA/DHA and type 2 diabetes risk have produced contradictory results. The positive association observed between EPA/DHA and type 2 diabetes risk in our study is consistent with findings from previous cohort studies that examined dietary n-3 PUFA and type 2 diabetes risk [7], [31]. While another investigation of fatty acid biomarkers observed a lower risk of type 2 diabetes with increased plasma EPA/DHA concentration [3], finding of a recent meta-analysis of cohort studies show no association between dietary EPA/DHA and type 2 diabetes risk [32]. The difference in risk observed between these studies may be due to the vulnerability of dietary n-3PUFA to oxidative damage; this may adversely affect insulin resistance and increase the risk of type 2 diabetes [33]. N-3PUFA may contribute to higher glucose concentrations through a number of mechanisms. It may increase hepatic gluconeogenesis [34] by increasing uptake and oxidation of free fatty acids in the liver [35] and lowering triacylglycerol [36], or it could lower glucose utilization and increase glucagon-stimulated C-peptide [37].

Lignoceric acid is primarily originates from endogenous synthesis by successive chain elongation of shorter chain SFA. In whole blood it is mainly located in the erythrocyte membranes. Elevated levels of fasting whole blood 24∶0 may be the result of its reduced degradation in the peroxisomes. The association of lignoceric acid with reduced type 2 diabetes risk observed in this study is a novel finding and merits further investigation.

The absence of a difference between fatty acid desaturase products in fasting whole blood of non-diabetic and type 2 diabetes suggests that endogenous fatty acid metabolism is not affected in type 2 diabetes patients. Previous studies, using animal models, have demonstrated an enhancement of Δ^9^-desaturase activity but no change in Δ^6^- and Δ^5^-desaturase activities [38]. It is likely that other factors such as age, duration of diabetes and dietary habits of the study participants interact to influence fatty acid metabolism resulting in no change overall.

To the best of our knowledge, only a few studies have used whole-blood fatty acids as a biomarker of intake [15], [39] and these studies investigated conditions other than type 2 diabetes. Fasting whole blood combines two different pools of fatty acids, the plasma and the erythrocytes, these pools have different half-lives as erythrocytes have a life-span of around 100–120 days and contain fatty acids that reflect longer term intake. It has been shown that fasting whole blood is a suitable biomarker of fatty acid intake; due to ease of collection, processing, and storage [15]. Our finding of no association between fasting whole blood concentration of total SFA and MUFAs with type 2 diabetes is not surprising as these two classes of fatty acids can be endogenously synthesized from carbohydrates [15], [40].

The major strengths of this study include the use of a nested case-control design where the cases emerge from a well-defined source population and the controls are sampled from the same predefined cohort. All incident cases in the cohort are compared to a random subset of community-dwelling participants who did not develop type 2 diabetes during the follow-up period of the parent cohort study.

Notwithstanding fasting whole blood combines two different pools of fatty acids, the plasma and the red blood cells, and thus is not as accurate indicator of long-term fatty acid intake as red blood cells alone. However, these pools have different half-lives and provide complementary information. Whole blood is also a convenient and easy to use source; and the use of fasting whole blood is likely to minimise the influence of recent dietary fat intake [15]. Furthermore, fasting whole blood fatty acid measurements were conducted on blood collected before the development of type 2 diabetes. This temporality strengthens the argument for a causal association between fasting whole blood fatty acids and the development of type 2 diabetes. To ensure that all cases of type 2 diabetes were incident cases we excluded all participants with self-reported diagnosis of type 2 diabetes at baseline or fasting serum glucose ≥7.0 mmol/L). Limitations of this study should be also noted. There was no attempt to verify self-reported type 2 diabetes however self-report is a well-accepted measure of diabetes status in population-based epidemiological studies. Numerous other studies have demonstrated a high level of agreement between self-reported type 2 diabetes and more objective measures of type 2 diabetes status in different populations [41], [42], [43]. Further, there is a concern about the possibility of residual confounding. Considering that type 2 diabetes cases had a higher BMI and energy intake, which play a pivotal role in increased oxidative stress, the possibility that oxidative stress is casually related should be considered.

Collectively, this nested case-control study suggest that higher concentrations of fasting whole blood n-6PUFA (ARA and DGLA) and n-3PUFA (ALA, EPA, and DHA) were associated with an increased risk of diabetes, whereas increased fasting whole blood concentrations of lignoceric acid is inversely associated with diabetes risk in adults.
